# Healthcare Data-Based Prediction Algorithm for Potential Knee Joint Injury of Football Players

This article has been retracted.

**DOI:** 10.1155/2021/3461648

**Published:** 2021-11-24

**Authors:** Yue Yu, Zi Ye

**Affiliations:** The Ministry of Public Basic Course, Wuhan Institute of Design and Sciences, Wuhan 430205, China

## Abstract

It is important to predict the potential harm to the knee joint in order to prevent football players from inflicting numerous injuries to the knee during activity. Numerous professionals have been drawn to this subject, and many viable prediction systems have been developed. Prediction of potential knee joint injury is critical to effectively avoid knee joint injury during exercise. The current prediction algorithms are mainly implemented through expert interviews, medical reports, and historical documents. The algorithms have problems with low prediction accuracy or precision values. There is a need to understand more knee injury factors and improve the prediction accuracy; hence, the intelligent prediction algorithm for potential injury of knee joints of football players is proposed in this paper. Firstly, the characteristics of the knee joint injury and the injury factors of the football players are gathered and analyzed. Then, the damage is predicted by the similarity measurement. The experimental results show that the proposed algorithm has higher prediction accuracy and shorter time. According to the findings of a survey that collected healthcare data, several key factors contribute to football knee injuries. To a degree, this algorithm can predict the likelihood of a football player's knee injury.

## 1. Introduction

Football is known as the “world's first sport” and is deeply loved by the masses. However, due to the strong confrontation and competition of football and its popularization, the lack of scientific training and guidance is often easy to cause various injuries and strains of athletes [1]. The definition of sports injury refers to the various injuries that athletes have in the process of sport. The occurrence of sports injuries is closely related to athletes' sports training, athletes' sports techniques, athletes' sports tactics, and athletes' sports environment. It is mainly in the motor system of the human body but also includes the blood vessels and nervous system damage of the human body [2]. Football is one of the sports with the highest incidence of trauma. According to statistics, in addition to some ordinary abrasions, athletes' knee injury is the most common problem in football, which seriously affects the physiology of football players [3]. In football, the more common sports injuries are knee injuries, including athlete's tibia joint pain, football player's tendonitis, football player's sacral syndrome, football player's quadriceps tendinitis, and athlete's knee around bursitis. The cognitive risk of knee injury in football players refers to the difference between subjective cognition and the objective risk of football trainers' potential danger [4]. The prediction of the potential injury of the knee joint of a football player refers to the situation in which the individual athlete of the football player may have a negative result during the exercise and the degree of damage to the consequences [5]. The competitive energy of football players is seriously affected and restricted by sports injuries. Knee joint injury is one of the most common injuries but very crucial for players to play any game [6]. Football players are unable to perform due to knee injuries during training and competition [7]. Normal training and participation in the competition seriously hindered the normal play and promotion of the football players' competitive level. They may also result in the termination of the sports career due to excessive knee injuries. To prevent football players from causing various injuries to the knee during exercise, it is necessary to predict the potential damage of the knee joint. This issue has attracted the attention of many professionals and has adopted many feasible prediction algorithms.

Based on the healthcare data, an algorithm for predicting the potential injury of knee joints of football players is proposed in [8]. Firstly, the questionnaire surveys investigated 800 athletes in a football match. Then, the causes of knee injury in athletes in this football match are classified, summarized, and statistically analyzed. According to the analysis results, the prediction results of potential injuries of the knee joint are obtained. The experimental results show that the internal cause of knee joint injury in football is mainly the specificity of knee joint structure. The external factors are related to the level of the football player's own technical level, the strength of the athlete's protection consciousness, the amount of exercise of the athlete during the training, and the medical supervision of the athlete. The results of the questionnaire survey providing healthcare data indicate that the main factors of the knee injury of football players are as follows: the athletes' early warm-up preparation activities are insufficient, accounting for 89.6%; the technical movement of athletes is unreasonable, accounting for 84.5%; athletes' self-protection awareness is weak, accounting for 82.8%; athletes' self-protection awareness is weak, accounting for 82.8%; athletes are overloaded with the training, accounting for 78.9%, and sports venue factors account for 75.2%. Based on the above data analysis, the potential damage of football players' knee joints is predicted. This algorithm can predict the potential knee injury of football players to a certain extent. However, many other potential injuries have not been found, which is not conducive to the prevention and treatment of knee injury in the later period.

Literature [9] proposes a prediction algorithm for the potential injury of knee joints in football players. Firstly, a stratified cluster sampling method is used to conduct a questionnaire survey on the injury of 5,000 athletes in a national football match. The survey includes the gender of the athlete, the time of the athlete's injury, the location and type of the athlete's injury, and the cause of the damage. The survey results show that the injury rate of football players is 53.9%. The most common injury site of athletes is a knee injury. The most common types of knee injury are knee joint abrasion, knee sprains, knee contusion, and knee joint strain. The ratio of these injuries is relatively close, among which male football players have the most strain of 27.3%, and female athletes accounted for 26.9% of the main injuries. The main reason for a knee injury is insufficient warm-up preparation before the event, accounting for 57.5%. Athletes' technical mistakes account for 40.7%, and athletes' personal physique reasons account for 43.1%. According to the stratified cluster sampling survey data, the potential damage of the knee joint of football players is predicted. The algorithm has the problem of low prediction accuracy.

In literature [10], to predict the potential damage of the knee joint of football players, firstly, a longitudinal tracking survey of 200 football players in Shandong Province is conducted, and all knee injuries and athlete training conditions that affect athlete training are recorded. All athletes' knee injuries are diagnosed by professional orthopedic experts. The incidence of knee injury is counted, and the hazard ratio of knee joint incidence of athletes in different grades and years is compared. The statistical results show that 100 athletes suffered injuries to the knee joint during the game, including 27 acute trauma of the knee, 19 old knee injuries, and 11 knee strains. Moreover, the 43 knee injuries are 14 medial collateral ligament injuries, 4 posterolateral horn injuries, 8 knee meniscus injuries, 3 anterior cruciate ligament injuries, 2 posterior cruciate ligament injuries, 3 tibia strains, and 9 other damage to the joints. The algorithm is more comprehensive for analyzing knee injury of football players, but it has low efficiency in predicting potential damage.

Machine learning predictors, swarm intelligence algorithms, and evolutionary techniques have been evolved remarkably. They are used by the researchers to solve many problems, including NP-hard problems such as the Knapsack problem [11], scheduling of “*m*” jobs on “*n*” resources [12], travelling salesman problem [13], subset sum problem [14], and halting problem [15]. Deep and machine learning is also contributing to solving the real-world problems of prediction and classification [16, 17]. The evolution is still taking place, and the performance of the algorithms is improving day by day [18]. Aiming at the shortcomings of the existing prediction algorithms in the area of knee injury, an intelligent prediction algorithm for football players' knee joint potential damage is proposed. The experimental results show that the proposed algorithm can improve the prediction accuracy and provide prerequisites for preventing knee injury in football players.

To overcome the knee injury problems in the athletes, the algorithm is proposed for predicting the potential injury in football players. Various internal and external factors were discussed, which are the major cause of the injuries on the field, and the results were obtained after the complete survey that could help reduce damage through injuries.

## 2. Materials and Methods

### 2.1. Characteristics of Knee Joint Injury

Using the method of questionnaire survey and football network database analysis and video analysis, three-dimensional motion analysis technology is used to analyze the knee injury details and characteristics of football players. The specific process is described below.

According to the athlete's age, height, weight, type of knee injury, activity time, movement characteristics, prematch preparation, and other factors, the relevant questionnaire was designed. At the provincial scene of football matches in Shanghai and Guangdong, questionnaires are distributed, filled out, and recycled. A total of 200 questionnaires are distributed, and 188 are recovered, with a recovery rate of 94%. A total of 180 valid questionnaires are analyzed, with an effective rate of 90%. In the process of plane fixed-point shooting, the sports video materials of football players are obtained, and then the images are analyzed by professional simulation software. Combined with the factors inducing knee injury in athletes, the corresponding indicators are selected for correlation analysis. The test indicators are shown in Table 1.

According to the test indicators in Table 1, the actual measured football player's exercise data is processed by SPSS, and the statistical results are analyzed for differences. According to the statistical results of the questionnaire survey, there are 126 athletes with knee injuries and 54 without injuries, accounting for 70% and 30%, respectively. Among them, 60 people with meniscus injuries accounted for 48% of the total number of injuries. Twenty-seven percent of the patella is injured, 28 of the collateral ligaments are injured, and the proportion of patellofemoral softening is 3%. The details are shown in Figure 1.

It can be seen from Figure 1 that the knee injury of football players is mainly meniscus injury, followed by patella and collateral ligament injury.

According to nature, athletes' knee injuries can be divided into three types: acute injury, chronic injury, and acute to chronic injury. Acute injury to the knee is caused by direct or indirect violence [19]. In the process of frequent football players, training or competition, often doing some action leads to sudden injury. Chronic injury is an injury caused by excessive long-term overloading of the knee joint. If the acute injury is not handled properly, the injury is not treated promptly or the training is performed in advance if the old injury is not cured, and the acute injury is converted to chronic injury.

According to the statistical results in Table 2, it can be seen that chronic injury accounted for a large proportion of knee injuries, reaching 63%.

The degree of knee injury of football players can be divided into three types:

1. The athletes who are still able to train according to the training plan after an injury are called mild knee injuries;
2. Athletes who are unable to continue training according to the training plan within one week after the injury and who need to reduce or stop local activities are called moderate knee injuries;
3. Athletes who are completely unable to exercise more than one week after the injury are called severe knee injuries.

It can be seen from Tables 3 and 4 that most of the knee injuries of football players are mainly moderate injuries. Most of the knee injury of football players is classified as moderate injury. The more frequent the athlete's movement is and the longer the exercise time is, the more the pressure exerted on the knee joint is. The chances of injury to the knee joint of the athlete increase more. The degree of injury to the knee joint will also increase. To study the relationship between knee injury and the season of football players, 112 football players who participated in the questionnaire for knee injury are further investigated. The results are shown in Table 5.

According to the results in Table 5, among the 112 football players with knee injuries, the proportion of athletes injured in spring, summer, autumn, and winter accounted for 16%, 28.6%, 25%, and 30.4% of the total number of knee injuries. The results show that knee joint injury is more likely to occur in winter and summer. In winter, due to the cold weather, the athletes are not ready for activities. The skeletal muscles of football players, the central nervous system, and athletes are not fully mobilized, so it is easy to cause knee injury. In summer, due to the high temperature, football players are prone to sports fatigue, resulting in the inattention of the athletes. In this case, sports players are prone to knee injuries.

Table 6 shows the time distribution table of knee injuries of football players. According to the survey presented, the knee injury of football players is mainly occurring in the training period, in which the proportion of males is 30%, and the proportion of females is 22%.

As can be seen from Table 7, the highest probability of knee injury in football players is the competition arena, accounting for 54%. Since the competition arena is a platform that reflects the staged training results of football players and proves their self-worth, they are more excited, and the probability of knee joint damage increases. The second highest is the training ground, which accounts for 42%. In addition to competitive games, football players are actively attaining training most of the time. For long-term repetitive training, knee injury is also aggravated by the increase in athlete training time.

### 2.2. Factors that Cause Knee Injury

There are various major factors that cause injuries on the field. They may be internal or external. A complete survey is done, and results are analyzed to know the reasons for injuries. Common reasons were psychological disorders, improper training before the match, improper warm-up, or overstressed person. According to the questionnaire filled out by 112 football players, 86 of them considered that insufficient preparation activities are an important cause of knee injury, accounting for 76.8% of the total number. There are 10 people with unreasonable training loads and excessive physical fatigue, accounting for 8.9% of the total number of knee injuries. There are 4 people who were not fully relaxed, accounting for 7.1% of the total number of knee injuries. Body collision, self-protection awareness, and poor physical fitness are the main factor of knee injuries, each accounting for 1.8% of the total number of knee injuries. The rest lack targeted rehabilitation training, training, or competition against injuries, and the bad weather is not selected by football players, all of which are 0%. The proportion of other factors is shown in Table 8.

Through comparative analysis, the main factors leading to knee injuries of football players include the following: inadequate preparation activities, physical fatigue, and inadequate relaxation. To more comprehensively analyze the main causes of knee injury in football players and to accurately predict the potential injury of football players' knee joints, it is necessary to conduct questionnaires and on-site interviews for football players.

The preparation activity is the most basic body warm-up exercise before the football player starts running. Its purpose is to fully mobilize the nervous system and organs to meet the specific requirements of football training or competition [20]. Knee joint injury can result if the athlete lacks preparatory activities or if the athlete's preparation activities are unreasonable.

Table 9 reveals that out of the 112 football players surveyed for knee injuries, 71.4% of the football players have gradually recognized the importance of preparation activities for athlete training or competition. Exercise fatigue is a temporary reduction in the working capacity of the body. It can be restored to the level of the original organism after proper rest and reasonable adjustment. The improvement of exercise level is the virtuous cycle of exercise fatigue and recovery. Usually, exercise fatigue is a normal physiological phenomenon, but it is also one of the important causes of knee joint injury [20]. Excessive fatigue can have adverse effects on the body, causing athletes' physical skills to be impaired or damaged. After exercise fatigue, it is easy to cause movement deformation, decreased sensitivity, judgmental errors, distraction, muscle stiffness, and body disharmony, resulting in knee injury in athletes [21, 22]. Among the 46 knee injury football players surveyed, they have ignored the self-protection measures that should be mastered to prevent knee injuries, such as ice stretching and wearing protective gear.

In view of the problems in Table 10, it is necessary to strengthen the knowledge of football players' self-protection against knee injuries so that football players realize the importance of self-protection awareness and provide accurate data for predicting potential injury.

According to Table 11, 21.4% of the football players did not perform any treatment after knee injury; 67.9% were treated within 24 hours of the knee injury; 8.9% were treated 24 hours after the knee injury; 1.8% dealt with injuries within 48 hours. According to the above survey data, most football players can deal with knee joint injuries in a timely and conscious manner. The structure of the cause of knee injury in football players is shown in Figure 2. This structure discusses various internal and external causes which lead to the damage. It includes physical ability factor of an athlete and some are due to lack of proper training. These causes due to which injury happens are classified into various aspects, depending on the physical ability of the athlete and training methodology. It might be a psychological cause or some other miscellaneous reasons [23].

### 2.3. Prediction of Potential Injury

Assuming that the size of the template image *A* of the football player's knee joint is *M* × *N*, the formula for calculating the similarity (MCD distance) of the knee joint injury image *B* of any football player of the same size is

(1) $$\begin{array}{c} D\left(A,B\right)=\overset{M}{\underset{i=1}{\sum }}\overset{N}{\underset{j=1}{\sum }}R\left(A_{i,j},B_{i,j}\right), \end{array}$$

where *i* and *j* are two pixels in the knee joint injury image and *R*(*A*_*i*,*j*_, *B*_*i*,*j*_) means gray scale absolute difference of the knee joint injury image. They should meet the conditions as

(2) $$\begin{array}{c} R\left(A_{i,j},B_{i,j}\right)=\left\{\begin{array}{cc} 1, & \left|A_{i,j}-B_{i,j}\right|<T,\\ 0, & \text{others}, \end{array}\right. \end{array}$$

where *T* is the threshold of exercise intensity.

According to formula (2), the gray level absolute differences of the pixels corresponding to the images *A* and *B* are compared. If the absolute value error is smaller than the motion intensity threshold, the two points in the image are considered similar. If the gray level absolute difference of the corresponding pixel in the entire image area is smaller than the motion intensity threshold, then the similarity between *A* and *B* is high. According to formula (1), the MCD distance is used as the current matching degree to determine whether a template update is required. If the judgment result is that an update is needed, follow the below steps.

Using the basic idea of uniform sampling, some pixels are selected from images *A* and *B* by the same distribution instead of all other pixels for error calculation. Assume that 25 percent points are calculated and SAD is used as the matching criterion. The sampling point error calculation expression is as follows:

(3) $$\begin{array}{c} \frac{1}{4}:\text{SAD}\left(k\right)=\sum_{0}^{7}\overset{7}{\underset{0}{\sum }}\left|S_{0}\left(2i,2j\right)-S_{K}\left(2i,2j\right)\right|, \end{array}$$

where *S*_0_ means physical factors, *S*_*K*_ is technology, and *K* represents training intensity. Using the basic idea of central sampling, taking 25 percent of the center of the 16 × 16 moving image for calculation, the calculation of the sampling point error is as follows:

(4) $$\begin{array}{c} \frac{1}{4}:\text{SAD}\left(k\right)=\sum_{0}^{7}\overset{7}{\underset{0}{\sum }}\left|S_{0}\left(i+4,j+4\right)-S_{K}\left(i+4,j+4\right)\right|. \end{array}$$

The above uniform sampling and central sampling are combined as the moving image matching criterion, and the motion vector predictive value is obtained by the directed synthesis algorithm of the motion vector. They are combined in pairs, and the absolute values of their *x* component differences and the absolute values of the *y* component differences are summed. The similarity of the vectors is measured. The smaller the calculated value is, the more similar the motion vectors of the two football players are. Supposed that ${\bar{V}}_{a}=\left(x_{a},y_{a}\right)$, ${\bar{V}}_{b}=\left(x_{b},y_{b}\right)$, and ${\bar{V}}_{c}=\left(x_{c},y_{c}\right)$ are the three motion vectors of the adjacent blocks of the football player image, which can be obtained by computerization:

(5) $$\begin{array}{c} ab=\frac{x_{a}x_{b}+y_{a}y_{b}}{\sqrt{x_{b}^{2}+y_{b}^{2}}},\\ ac=\frac{x_{a}x_{c}+y_{a}y_{c}}{\sqrt{x_{c}^{2}+y_{c}^{2}}},\\ bc=\frac{x_{a}x_{c}+y_{a}y_{c}}{\sqrt{x_{b}^{2}+y_{b}^{2}}}. \end{array}$$

According to the above formula, the distances *ab*, *ac*, and *bc* between the three motion vectors of the football player are obtained. Their smallest value is selected as the two most similar motion vectors for football.

Using the characteristics of the motion direction and the intensity of the adjacent motion vectors, the average of the angles of the two most similar motion vectors is taken as the angle of the predicted vector of the potential injury of the knee joint. The average of the modes of the two most similar motion vectors is taken as the modulus of the injury prediction vector. Through the calculation and simplification, the scaling factor of the potential injury of the knee joint in football players can be obtained:

(6) $$\begin{array}{c} \alpha =\frac{\sqrt{x_{a}^{2}+y_{a}^{2}}+\sqrt{x_{b}^{2}+y_{b}^{2}}}{2\sqrt{{\left(x_{a}+y_{b}\right)}^{2}}+\sqrt{{\left(x_{a}+y_{b}\right)}^{2}}}. \end{array}$$

The sports vector of the football player is as follows:

(7) $$\begin{array}{c} \overset{⟶}{V}=\alpha \left(\left(x_{a}+x_{b}\right),\left(y_{a},y_{b}\right)\right). \end{array}$$

Equation (7) is the case where the predicted vectors of the knee injury of the closest football players are ${\overset{⟶}{V}}_{a}$, ${\overset{⟶}{V}}_{b}$, and so on.

## 3. Results

The experiment uses two CASIO FH25 cameras with a high-speed animation shooting function produced in Japan to shoot football players in real time. The specific shooting parameters are set as follows: shutter speed is 1/2000 s; shooting aperture is F3.4; shooting focal length is 92 mm; and shooting frequency is 120 fps (640 ∗ 480). The experiment utilizes two tripods. The operation setting is as follows: the height of the camera tripod is 1.5 m and the camera tripod is calibrated to maintain the level. When shooting the overall movement of the football player, the height of the camera is roughly the same as that of the athlete's hip. The video and image data obtained by the shooting are made by the APAS video analysis software produced in the United States, and the operation steps are as follows: the knee player's knee flexion action on the training field is selected for analysis and processing. In the process of motion video analysis, the Japanese Matsui Shoji human body parameter model was tested, and six knee joint points were selected as the quantization points according to the standard of the football player human body model. The 3D data of the football player is smoothed by the low-pass filtering method, the cutoff frequency of the motion video is selected to be 16 Hz, and the obtained raw data of the football player is saved in Excel. The size of the training intensity is an important factor in the potential injury of the knee joint of the athlete. The probability of knee joint injury caused by the weekly training intensity of football players is analyzed by survey analysis. The results are shown in Figure 3.

According to Figure 3, when the training intensity of the football player is one time a week, the probability of actual injury of the knee joint of the athlete is less than 10%. When the training intensity of football players is 2 times a week, the probability of actual injury of the athlete's knee joint is 20%. When the training intensity of football players reaches 5 times a week, the probability of actual injury of the athlete's knee joint is 45%. When the training intensity of football players reaches 8 times a week, the probability of actual injury to the knee joint of the athlete reaches 90%. Based on the above analysis, the greater the training intensity of football players is, the greater the actual probability of knee joint injury is. When the weekly training intensity is greater than or equal to 8 times, it means that the knee joint must be damaged.

During the training or competition, the knee injury caused by different knee angles is also different. The experimental results are shown in Figure 4. It can be seen from Figure 2 that the probability of knee joint loss increases with the increasing knee angle of football players. When the knee angle is 10 degrees, the probability of knee injury is less than 15%; when the angle is 30 degrees, the probability of damage is 32%; when the knee angle reaches 80 degrees, the probability of knee injury reaches about 80%.

As can be seen from Figures 3 and 4, the probability of knee joint injury of football players is closely related to the training intensity and the knee angle of the athlete. In order to achieve accurate prediction of injury, it is necessary to control the training intensity and knee angle of the football player.

The accuracy of the injury prediction is a measure of whether the potential injury of the knee joint of the football player will occur. The expression is

(8) $$\begin{array}{c} \text{Accuracy of injury prediction}=\frac{\text{prediction injury person}}{\text{actural injury person}}\times 100\%. \end{array}$$

According to the above formula, the prediction accuracy of the three algorithms is compared and analyzed, and the results are shown in Figure 5.

Figure 5 shows the relation between the number of football players surveyed per person to the predictive accuracy of a potential knee injury. It is clear from Figure 5 that, for the same number of players, the paper algorithm shows a maximum chance of injury. It can be seen from Figure 5 that the algorithm presented in [19] has the lowest prediction accuracy for the potential injury of the knee joint in football players; the prediction accuracy of the proposed algorithm is the highest. This is due to the incomplete analysis of the intrinsic and extrinsic factors of knee joint injury by the other two contrast algorithms. The algorithm of this paper comprehensively analyzes the characteristics of knee injury and the cause of injury in football players, so the prediction accuracy is the highest. The time consumption of the predicted injury of the three algorithms is compared and analyzed, and the results are shown in Figure 6.

It is the graph of the number of football players surveyed per person to the time consumed for the prediction of potential knee joint injury per second. It is clear that the algorithm proposed by this paper shows maximum efficiency and is result-oriented. According to Figure 6, it can be seen that when the number of football players participating in the survey increased to 19, the prediction time consumption of the literature [18] algorithm showed a rapid growth trend. After the number of football players participating in the survey increased to 10, the prediction time of the literature [19] algorithm tends to be stable and stabilizes at around 46 s. Throughout the experiment, the prediction time consumption of the algorithm is at a low level, and the average time is about 13 s. It can be seen that compared with the other two algorithms, the prediction of the proposed algorithm takes less time and has superior performance.

## 4. Discussions

In the MATLAB 7.0 environment, the intelligent prediction platform of football player's knee joint potential injury is built. The cloud computing platform is a six-core AMD Ryzen 5 1600X processor. The training intensity of football players and the influence of different knee flexion angles on knee joint injuries are analyzed, and both are positively correlated with knee joint injuries. To fully prove the effectiveness of the proposed algorithm, the prediction accuracy and time consumption are selected as the comparison indicators, and the algorithms of [18, 19] are compared and analyzed. The experimental results show that the prediction accuracy of the proposed algorithm is much higher than the others, and it takes less time and better performance.

## 5. Conclusions

To prevent football players from causing various injuries to the knee during exercise, it is necessary to predict the potential damage of the knee joint. The traditional algorithm is used to predict the potential damage of the knee joint, the analysis of the injury factor is not comprehensive, and the prediction accuracy is low. An intelligent algorithm is predicted for a football player's knee joint. The survey results providing healthcare data discussed the major reasons for this damage. There are internal and external reasons. The proposed algorithm consumes optimal time as shown in results for predicting the outcome of knee injury and outperforms other predicting techniques taken for comparative study. The predictive accuracy of the proposed algorithm is highest as compare to other predictive models of knee injury. The experimental results show that the proposed algorithm can improve the prediction accuracy and provide prerequisites for the prevention of knee injury in football players. Also, the training intensity and knee flexion angle affect the knee joint injury probability of football players, and the proposed algorithm has higher prediction accuracy and shorter prediction time, which lays the foundation for the subsequent prevention of knee injury of football players. This algorithm can predict the likelihood of a football player's knee injury to a degree, but there are still many additional potential ailments that have yet to be discovered, making it difficult to prevent and treat knee injuries in the future.

## Figures and Tables

**Figure 1:** The proportion of the type of knee injury in football players.

**Figure 2:** The structure of the cause of knee injury in football players.

**Figure 3:** Effect of training intensity on knee joint injury.

**Figure 4:** Effect of different knee angles on knee joint injury.

**Figure 5:** Predictive accuracy of different algorithms.

**Figure 6:** Prediction time consumption of different algorithms.

**Table 1:** Football players knee joint injury indicators.

Biomechanical kinematics of knee joint injury in football players	Football player's physical special qualities
Center of gravity	Speed endurance
Knee speed	Strength endurance
Knee angular velocity	
Knee flexion angle	Speed sensitivity

**Table 2:** Survey results of knee joint injury properties.

Knee joint injury properties	
Acute injury	30 persons (24%)
Chronic injury	80 persons (63%)
Acute to chronic injury	16 persons (13%)

**Table 3:** Survey results of the degree of knee injury in football players.

Degree of knee injury	
Mild injury	30 persons (24%)
Moderate injury	90 persons (71%)
Severe injury	6 persons (5%)

**Table 4:** Survey results of the relationship between knee injury degree and exercise time.

Degree of knee injury	Exercise time
Mild injury (30 persons)	1-2 times/week, 3–6 h/time (8 persons, 27%)
	7–9 times/week, 3–6 h/time (22 persons, 73%)
Moderate injury	1-2 time/week, 3–6 h/time (14 persons, 16%)
	7–9 time/week, 3–6 h/time (38 persons, 84%)

**Table 5:** Survey results of the relationship between season and knee joint injury (*N* = 112).

Season	Spring	Summer	Autumn	Winter	Total
Number of athletes	18	32	28	34	112
Proportion (%)	16	28.6	25	30.4	100

**Table 6:** Time distribution table of knee injuries of football players.

Time gender	Before training		In training		After training		Actual combat and competition	
	Male	Female	Male	Female	Male	Female	Male	Female
Person	4	6	30	22	4	4	16	14
Percentage (%)	4	6	30	22	4	4	16	14

**Table 7:** Survey of knee injury sites of football players.

Site	Training ground	Competition arena	Amateur activity field	Others
Person	42	54	2	2
Percentage (%)	42	54	2	2

**Table 8:** Survey results of the causes of knee injury in football players (*N* = 112).

Technical action	No. of persons	Percentage (%)
Insufficient preparation activities	86	76.8
Incomplete relaxation	8	7.1
Physical fatigue	10	8.9
Body collision	2	1.8
Poor sense of self-protection	2	1.8
Poor physical fitness	2	1.8
Sport equipment	2	1.8
Targeted rehabilitation training	0	0
Injury training or participate in competitions	0	0
Bad climate factor	0	0

**Table 9:** Survey of targeted preparation activities and collation activities (*N* = 112).

	Yes	No	Total
Person	80	32	112
Percentage (%)	71.4	28.6	100

**Table 10:** Survey results of football players' self-protection awareness (*N* = 46).

Self-protection awareness	No. of persons	Total (%)
Self-processing ability	12	26
Ice	9	19.5
Stretching	5	10.9
Wearing protective gear	20	43.5

**Table 11:** Treatment of football players after knee joint injury (*N* = 112).

	Without treatment	Within 24 h	After 24 h	After 48 h	After 72 h	Total
Number	24	76	10	2	0	112
Percentage (%)	21.4	67.9	8.9	1.8	0	100

## Data Availability

Data will be made available on request.
